# Evaluation of Nursing Effects of Pelvic Floor Muscle Rehabilitation Exercise on Gastrointestinal Tract Rectal Cancer Patients Receiving Anus-preserving Operation by Intelligent Algorithm-based Magnetic Resonance Imaging

**DOI:** 10.1155/2022/1613632

**Published:** 2022-05-19

**Authors:** Lijuan Zhang, Feng Wang

**Affiliations:** ^1^Department of Gastroenterology, Shanxi Province Cancer Hospital/Shanxi Hospital Affiliated to Cancer Hospital, Chinese Academy of Medical Sciences/Cancer Hospital Affiliated to Shanxi Medical University, Taiyuan 030013, Shanxi, China; ^2^Clinical Laboratory, Shanxi Children's Hospital, Taiyuan 030013, Shanxi, China

## Abstract

Based on magnetic resonance imaging (MRI) technology under artificial intelligence algorithm, the postoperative nursing effects of pelvic floor muscle rehabilitation exercise on gastrointestinal tract rectal cancer (RC) patients were investigated. A total of 88 patients receiving RC anus-preserving surgery in hospital were selected. The included patients were divided randomly into the experimental group (44 cases) and the control group (44 cases). Patients in the control group engaged in Kegel motion, while patients in the experimental group underwent self-designed comprehensive pelvic floor training. Anorectum function rating scale and quality of life questionnaire for colorectal cancer (EORTC QLQ-CR29) were utilized to compare and analyze anus functions and living quality of patients in the two groups. Besides, all patients in two groups received MRI examinations, and images were processed by a convolutional neural network (CNN) algorithm. The results showed that in MRI images, there were significant signal differences between lesion tissues and normal tissues. After being processed by an artificial intelligence algorithm, the definition of MRI images was remarkably enhanced with clearer lesion edges. The quality of images was also significantly improved. Besides, the comparison of anus functions of patients in two groups showed that the differences demonstrated statistical meaning after the intervention (*P* < 0.05). In conclusion, artificial intelligence algorithm-based MRI and comprehensive pelvic floor muscle exercise showed significant application prospects and values in the recovery of patients' intestinal functions after RC anus-preserving surgery.

## 1. Introduction

Rectal cancer (RC) is one of the most common malignant tumors and one of the most significant causes of death by cancer at present. Relevant statistics show that the incidence of RC is ranked in the 3^rd^ place among cancers and the 5^th^ place in mortality among cancers in China [1, 2]. At present, there is still no consensus on its pathogenesis, which may be due to heredity, environmental factors, and dietary habits [3]. Surgical treatment is the main therapeutic method of the disease [4]. However, anus-preserving is difficult in the surgical operations of RC because most tumors are located at the base of the pelvic floor and close to dentate lines. In recent years, anastomotic and surgical technologies are continuously developed and improved, and neoadjuvant therapy as well as total mesorectal excision (TME) are gradually proposed [5, 6]. RC anus-preserving surgery becomes the main method of treating RC gradually. The method saves many patients from carrying pockets for whole life. However, various intestinal dysfunctions and mental dysfunctions occur after surgery. As a result, the incidence of these symptoms seriously affects patients' living quality [7]. Although sphincter functions are completely preserved by RC anus-preserving surgery, intestinal anatomical structure and functions are impaired and disturbed in tumor excision. In addition, most patients suffer from multiple intestinal symptoms after surgery because of radiotherapy and other factors. According to considerable clinical data, about 50% to 90% of patients suffer from postoperative low anterior resection syndrome (LARS) [8, 9]. After the surgery, early symptoms are very significant with high incidence. However, these symptoms will probably last for a lifetime if treatment and recovery measures are not taken in time [10, 11]. At present, the common nursing methods include transanal irrigation, electrical stimulation of sacral nerves, biofeedback therapy, rectal balloon training, and Kegel motion [12, 13]. Foreign relevant studies are carried out at an earlier time, and most of them focus on the recovery of patients' intestinal functions by combining multiple training methods [14]. The improvement of patients' incontinence is also focused. In contrast, patients' living quality and other common symptoms are less focused. There is still no rehabilitation nursing method regarded as effective by the public. In addition, extensive and multi-center experimental validation is inadequate in most studies. Generally speaking, the scientificalness and safety of pelvic floor muscle training after RC anus-preserving surgery needed to be further verified and studied [15].

In recent years, imaging technology has constantly improved; RC diagnosis and therapeutic effect assessment methods have become more diversified gradually. Currently, the main assessment methods of diagnostic and therapeutic effects on RC include endorectal ultrasonography (ERUS), computed tomography (CT), and magnetic resonance imaging (MRI). For example, some scholars used MRI for the diagnosis of RC patients and an analysis of their diagnostic efficiency. The results showed that the accuracy, sensitivity, and specificity of MRI in diagnosing RC were 92%, 90%, and 85%, respectively. MRI has become the main method of clinical RC diagnosis. The extraction of effective features from numerous medical images is the focus of present studies to provide the basis for clinical diagnosis and treatment. The feature expression ability of traditional learning algorithms is weak because of their shallow training model level. As a result, the application of traditional learning algorithms is restricted in medical image feature extraction. On the contrary, deep learning algorithms make up for the defects of traditional learning algorithms [16]. In particular, the deep convolutional neural network (CNN) algorithm is a method with the most significant research values and potential in image processing and analysis. Furthermore, a large amount of research data demonstrates that the error rate of feature recognition is reduced to 3.5% [17]. To sum up, deep CNN shows significant advantages and application prospects in imaging processing and feature extraction. Nowadays, there are many studies on the application of CNN in medical imaging, including image segmentation, image classification, image registration, and target detection [18].

On the grounds of the previous researches, a set of pelvic floor muscle exercise methods was designed independently. Besides, artificial intelligence algorithm-based MRI technology was utilized to discuss postoperative recovery therapeutic effects of the method on RC patients receiving anus-preserving surgery, which aimed to provide new ideas and a reference basis for the diagnosis, treatment, and postoperative recovery of clinically relevant diseases.

## 2. Materials and Methods

### 2.1. Research Objects

A total of 88 patients receiving RC anus-preserving surgery in hospital between March 2019 and November 2020 were selected, including 58 male patients and 30 female patients. The average age of the included patients was 55.3 ± 11.3 years old, and they were divided randomly into the experimental group (44 cases) and the control group (44 cases). All the included patients had signed the informed consent forms and this research had been approved by the ethics committee of the hospital.

Inclusion criteria: patients who were diagnosed with RC by colonoscopy or pathological examination and the distance between the lower edge of the patient's tumors and dentate lines was equal to or shorter than 10 cm. Patients who accepted RC radical excision with anal sphincter retained. Patients who volunteered to engage in the research.

Exclusion criteria: patients who suffered from temporary or permanent stoma; patients who had anastomotic leak and other severe complications. Patients who got other complicated intestinal functional diseases before surgery, such as irritable bowel syndrome, Crohn's disease, and ulcerative colitis. Patients who took drugs that affected intestinal functions over 3 weeks within 1 month before surgery, such as antidiarrheal agents, laxatives, and morphine. Patients who received the auxiliary treatments of other intestinal functions imaging, such as biofeedback therapy. Patients who received the surgical treatment of other intestinal functions imaging, such as anorectal surgery, pelvic surgery, abdominal surgery, and spinal surgery. Patients who suffered from mental diseases. Patients who suffered from complications of severe heart, lung, kidney, and musculoskeletal diseases.

### 2.2. Postoperative Nursing Methods

Patients in both groups were offered medication, diet, and life guidance. Besides, they were also provided with anus peripheral skin care, anastomotic stoma expansion, regular defecation training, and other conventional nursing measures. Based on the above guidance and nursing measures, pelvic floor muscle rehabilitation training was carried out 1 week after postoperative defecation. Specific exercise intervention methods were as follows.

In the control group, patients were instructed to perform the Kegel motion. Before the exercise, patients were asked to empty their urinary bladders. After that, they needed to take a comfortable position, such as lying on their back or sitting. Patients should try to keep their leg, abdomen, and back muscles as relaxed as possible, and try their best to squeeze perineal muscles upward and inward until pelvic muscles and levator ani muscles were lifted upward. The squeezing action needed to be kept for 5 seconds, and then patients relaxed for 10 seconds. The above steps constituted a group of exercises. A total of 10 groups of exercises needed to be performed for each time. Each single exercise lasted for about 3 minutes and was performed 3 times each day.

In the experimental group, the training methods were improved and integrated based on considerable literature and data as well as the advice offered by anorectal surgery experts, rehabilitation therapists, and anorectal surgery nursing staff. The contents of the training included abdominal respiration, abdominal massage, Kegel motion, cross-leg anus lifting motion, and bridging anus lifting motion.  Table 1 shows specific exercise methods below. Each single exercise lasted for 8 to 10 minutes, 3 times each day.

### 2.3. Observation Indexes

Patients' general data included social demography data (age, gender, education level, economic income, and payment methods of medical expenditure) and disease-related data (tumor differentiation levels, medical history, and surgical methods).

In terms of the anorectum function rating scale, the evaluation contents of the scale included defecation intention, defecation control, defecation sensory functions, defecation times, and defecation time. Each of the above five aspects included 3 levels, and each level was assigned with 0, 1, and 2 points, respectively. The total points for each level ranged from 0 to 10. Based on the general evaluations in five aspects, the anus functions were divided into four levels, including excellent level (9–10 points), good level (7–8 points), intermediate level (5–6 points), and poor level (0–4 points). Besides, excellent and good level rate = (excellent level rate + good level rate)/total number of cases  ×  100%.

The quality of life questionnaire for colorectal cancer (EORTC QLQ-CR29) included four aspects of body image: anxiety, weight, and sexual desire. Four aspects included a total of 19 items. In each item, there were four levels of answers which were none, a little, a lot, and quite a lot. The four levels corresponded to 1, 2, 3, and 4 points, respectively. The scoring method was polarization method.

### 2.4. Examination Methods

A Philips superconductive nuclear magnetic resonance instrument (Prodiva 1.5 T, No. 82307) was adopted with phased-array surface coils. Sagittal, axial, and coronal scanning were performed. The slice thickness was 4 mm without spacing. Before the examination, no intestinal preparation was required. During the examination, patients needed to take a supine position. The center of the surface coil was placed at the pubis symphysis. Besides, the middle axial slice should be kept perpendicular to the anal tubes, and sagittal and coronal slices needed to be balanced with the anorectal axis during the scanning. During the examination, patients needed to breathe calmly and minimize body movement as well.  Table 2 demonstrated specific scanning parameters below.

### 2.5. Image Processing Methods

The denoising process was as follows. The array with *f*(*x*, *y*) of the image being *M*×*N* was processed, and the image was *g*(*x*, *y*). The gray level of the images was determined by the average value of the gray levels of several pixels including the field (*x*, *y*). The processed image is expressed by the following equation:

(1) $$\begin{array}{c} g\left(x,y\right)=\frac{1}{M}\sum_{\left(i,j\right)\in s}f\left(i,j\right). \end{array}$$

In the above equation, *x*, *y* = 0, 1, 2, ..., *N*-1, *S* denoted the field collection with the point (*x*, *y*) as the center, and *M* referred to the total number of coordinate points in *S*. In terms of multiple images, the original image was set to be *f*(*x*, *y*) and image noise was *n*(*x*, *y*). Then, the noisy image g(*x*, *y*) is expressed by the following equation:

(2) $$\begin{array}{c} g\left(x,y\right)=f\left(x,y\right)+n\left(x,y\right). \end{array}$$

If noises were unrelated and the average value was 0, the equation generated is as follows:

(3) $$\begin{array}{c} f\left(x,y\right)=E\left[g\left(x,y\right)\right]. \end{array}$$

In the below equation, *Eg*[(*x*, *y*)] represented the expected value of *g*(*x*, *y*), and *M* noisy images were averaged to generate the following equations:

(4) $$\begin{array}{c} f\left(x,y\right)=E\left[g\left(x,y\right)\right]∼\overset{-}{g}\left(x,y\right) \end{array}$$

(5) $$\begin{array}{c} \delta_{g\left(x,y\right)}^{2}=\frac{1}{M}\delta_{n\left(x,y\right)}^{2}. \end{array}$$

In the above two equations, $\delta_{\bar{g}\left(x,y\right)}^{2}$ and *δ*_*n*(*x*, *y*)_^2^ were the variances of $\overset{\text{\_}}{g}$ and *n* at the point (*x*, *y*).

The equations adopted for the edge detection process are as follows:

(6) $$\begin{array}{c} \psi^{1}\left(x\right)=\frac{\text{d}\theta \left(x\right)}{\text{d}x},\\ \psi^{2}\left(x\right)=\frac{{\text{d}}^{2}\theta \left(x\right)}{\text{d}x^{2}}. \end{array}$$

(7) $$\begin{array}{c} w^{1}f\left(s,x\right)=f*\psi_{s}^{1}\left(x\right),\\ w^{2}f\left(s,x\right)=f*\psi_{s}^{2}\left(x\right).\\ =s\frac{\text{d}}{\text{d}x}\left(f*\theta_{s}\right)\left(x\right).\\ =s^{2}\frac{{\text{d}}^{2}}{\text{d}x^{2}}\left(f*\theta_{s}\right)\left(x\right). \end{array}$$

(8) $$\begin{array}{c} w^{1}f\left(s,x\right)=f*\left(s\frac{d\theta_{s}}{dx}\right)\left(x\right)\\ =s\frac{\text{d}}{\text{d}x}\left(f*\theta_{s}\right)\left(x\right).\\ =s^{2}\frac{{\text{d}}^{2}}{\text{d}x^{2}}\left(f*\theta_{s}\right)\left(x\right). \end{array}$$

(9) $$\begin{array}{c} w^{2}f\left(s,x\right)=f*\left(s^{2}\frac{d^{2}\theta_{s}}{dx^{2}}\right)\left(x\right)\\ =s^{2}\frac{{\text{d}}^{2}}{\text{d}x^{2}}\left(f*\theta_{s}\right)\left(x\right). \end{array}$$

The membrane value of discrete binary wavelet transform *W*_2^*j*^_^1,*d*^*f*(*n*, *m*), *W*_2^*j*^_^2,*d*^*f*(*n*, *m*) of point (*n*, *m*) is expressed by the following equation:

(10) $$\begin{array}{c} M_{2^{j}}^{d}f\left(n,m\right)=\sqrt{{\left|W_{2^{j}}^{1,d}f\left(n,m\right)\right|}^{2}+{\left|W_{2^{j}}^{2,d}f\left(n,m\right)\right|}^{2}}. \end{array}$$

The phase angle is expressed as follows:

(11) $$\begin{array}{c} A_{2^{j}}^{d}f\left(n,m\right)=\text{arg tan}\left(\frac{W_{2^{j}}^{2,d}f\left(n,m\right)}{W_{2^{j}}^{1,d}f\left(n,m\right)}\right). \end{array}$$

### 2.6. Statistical Analysis

The analysis of all the data was completed by the statistical product and service solution SPSS 19.0. Measurement data were expressed by the mean +standard deviation and tested by an independent sample *t*-test. The comparison of enumeration data was completed by the chi-square test. *P* < 0.05 indicated that the differences showed statistical significance.

## 3. Results

### 3.1. Patients' General Data

Table 3 shows patients' general data below. According to Table 3, the differences in age, gender, tumor differentiation, and anal edge tumor height of patients in the two groups demonstrated no statistical significance (*P* > 0.05).

### 3.2. Intelligent Algorithm-Based MRI Processing

Figure 1 displays MRI images of typical cases before and after the processing by an artificial intelligence algorithm. In Figure 1, the images were of Case 1, Case 2, Case 3, and Case 4, respectively, from left to right, and the scanning positions were sagittal, axial, coronal, and sagittal positions, respectively. The analysis of Figure 1 demonstrated that there were significant signal differences between lesion tissues and normal tissues in MRI images. After the processing by an artificial intelligence algorithm, the definition of MRI images was remarkably enhanced with clearer lesion edges. Obviously, image quality was also significantly improved.

### 3.3. Comparison of Anus Functions of Patients in Two Groups before and after Intervention

Figure 2 displays the results of the comparison of anus functions of patients in two groups before the intervention. The analysis of Figure 2 revealed that the number of patients with excellent, good, intermediate, and poor levels of anus functions was 3, 9, 20, and 12, respectively, in the experimental group before the intervention. The excellent and good level rate reached 27%. In the control group, the number of patients with excellent, good, intermediate, and poor levels of anus functions was 1, 8, 22, and 13, respectively, and the excellent and good rates amounted to 20%. The comparison of anus functions in the two groups before the intervention showed no statistical significance (*P* > 0.05).

Figure 3 shows the comparison results of the anus functions of patients in two groups after the intervention. Figure 3 demonstrated that the number of patients with excellent, good, intermediate, and poor levels of anus functions in the experimental group 3 months after the intervention was 16, 22, 2, and 4, respectively. The excellent and good rates reached 86%. In the control group, the number of patients with excellent, good, intermediate, and poor levels of anus functions was 6, 20, 13, and 5, respectively, and the excellent and good rate amounted to 59%. After the intervention, the comparison of anus functions between two groups showed statistical significance (*P* > 0.05).

### 3.4. Comparison of Living Quality of Patients in Two Groups before and after Intervention

Figure 4 displays the comparison results of living quality of patients in two groups before the intervention. It was demonstrated in Figure 4(a) that the comparison of the score of each item in living quality between the experimental group and the control group before the intervention showed no significant difference. Besides, the comparison between groups showed no Figure 4(b) statistical significance as well (*P* > 0.05). The above results indicated that the data of two groups were comparable.

### 3.5. Comparison of Living Quality of Patients in Two Groups after Intervention

Figure 5 illustrates the comparison results of the living quality of patients in two groups after the intervention.  Figure 5(a) revealed that some symptoms of patients in the experimental group were significantly improved 3 months after the intervention, including (Figure 5(b)) frequent urination, defecate frequency, abdominal distension, dry mouth, fecal incontinence, and anus peripheral skin pain. The comparison of the scores in the above items showed significant differences and statistical meaning between the experimental group and the control group (*P* < 0.05).

## 4. Discussion

RC is defined as malignant tumors appearing in the intestinal tracts about 15 cm away from the anal edges, and it is one of the main death causes related to cancers at present. Both the incidence and mortality of RC in cities are higher than those in rural areas, and the incidence and mortality of RC among males were higher than those among females as well [19]. In the early phase, there are usually no significant clinical symptoms. Defecation habits of patients are often changed in the middle phase of RC, such as slenderer or flatter stools. Some patients suffer from defecation frequency, tenesmus, anus discomfort, and hypogastrium pain [20]. At an advanced phase, bloody stool or mucus usually appears. If tumors further spread to the prostate, some complications of urethral stimulus will occur, such as frequent urination, urgent urination, dysuria, and hematuria [21]. Although traditional surgical treatment methods can radically cure tumors, it is usually difficult to retain an anus because of the short distance from dentate lines. As a result, patients need to carry pockets for their lifetime, which seriously reduces patients' living quality.

With the continuous development of adjuvant therapy and anastomat in recent years, anus-preserving surgery can not only radically cure RC but also can retain anus successfully. This surgery addresses the problems with traditional surgical methods and greatly improves patients' living quality [22]. According to relevant studies, the above symptoms of some patients will be alleviated 1 to 2 years after RC anus-preserving surgical treatment. However, the symptoms will last for a lifetime among most patients, which causes great damage to patients both psychologically and physically [23]. Hence, it is indispensable to carry out some pelvic floor muscle rehabilitation training to help patients recover their intestinal functions. The impacts of pelvic floor muscle rehabilitation training on the postoperative living quality of RC surgical patients were investigated, and the results showed that it could obviously improve patients' postoperative anus functions and living quality. Consequently, the results provided the reference for the improvement of RC patient prognosis. In this work, a comprehensive pelvic floor muscle rehabilitation training program was raised on the basis of reviewing a large number of literatures. As the training was applied to the postoperative recovery of patients with RC anus-preserving surgery, the results were analyzed. The scores of anal functions and living quality in the experimental group were higher than those in the control group. This suggested that the postoperative pelvic floor muscle rehabilitation training was beneficial to postoperative functional recovery and to reducing complications, which was consistent with the results of previous related studies.

In RC diagnosis and therapeutic effect judgment, ERUS, CT, and MRI are all main examination methods. MRI shows a high resolution of soft tissues and multiplane imaging capacity. As a result, it can recognize tumors and peripheral tissues accurately and has become one of the main methods for diagnosing RC. With the continuous improvement of imaging technology, the quality requirements of medical images get higher and higher. Besides, computer technology is also developed widely in medicine, with the processing of medical images as a significant branch [24]. The deep learning algorithm is the most concerned and promising algorithm, and also a CNN algorithm that can make up for the defects of traditional algorithms. In addition, it shows extremely significant advantages in image processing and feature extraction [25]. Artificial intelligence algorithm-based MRI technology was utilized to evaluate the therapeutic effects of this deep learning algorithm. There were obvious differences in MRI images processed by an artificial intelligence algorithm of RC patients between tumors and peripheral tissues, and the quality of processed images was remarkably improved compared with that of the images to be processed. The differences indicated that artificial intelligence algorithm-based MRI showed significant application values and prospects in RC diagnosis and therapeutic effect assessment. MRI technology under an artificial intelligence algorithm was used for diagnosis and image processing of RC patients. The research results proved that the quality of processed MRI images was notably improved, the lesions were more prominent, and the boundary between the normal tissues and the lesions became clearer. It was illustrated that the method proposed in this work had a great application prospect in the diagnosis of RC.

## 5. Conclusion

Based on the reference to considerable literature, a comprehensive pelvic floor muscle training plan was proposed, and its therapeutic effects were evaluated by artificial intelligence algorithm-based MRI technology. The results demonstrated that there were obvious differences between MRI image tumors processed by an artificial intelligence algorithm of RC patients and peripheral tissues, and the quality of processed images was remarkably improved compared with that of the images to be processed. The differences revealed that artificial intelligence algorithm-based MRI showed significant application values and prospects in RC diagnosis and therapeutic effect assessment. What's more, the scores of anus functions and living quality of patients in the experimental group were both remarkably improved compared with those of patients in the control group after 3-month treatment.

## Figures and Tables

**Figure 1:** MRI images of typical cases.

**Figure 2:** Comparison results of anus functions of patients in two groups before intervention. ^*∗*^ Comparison to the control group, (*P*) < 0.05.

**Figure 3:** Comparison of anus functions of patients in two groups after intervention. ^*∗*^ Comparison to the control group, (*P*) < 0.05.

**Figure 4:** Comparison of living quality of patients in two groups before intervention. (a) function items; (b) symptoms.

**Figure 5:** Comparison of living quality of patients in two groups after intervention: (a) function items; (b) symptoms. ^*∗*^ Comparison to control group, (*P*) < 0.05.

**Table 1:** Training plan of comprehensive pelvic floor muscle exercise in the experimental group.

Training order	Training items	Training methods
Part 1	Abdominal respiration	Patients were instructed to place hands on abdomen, and keep abdominal muscles relaxed as they inhaled. After that, they were allowed to pause for 1 to 2 seconds. As they exhaled, abdominal muscles were contracted with the hands on abdomen declining. Each group of training lasted for 5 seconds and 5 groups of training needed to be completed every time.

Part 2	Abdominal massage	Patients were asked to lie on their backs and press tianshu, qihai, and guanyuan acupuncture points successively. Each acupuncture point was pressed by the thumbs for 1 minute. When the acupuncture points become swollen and get fever, the degree of pressure should remain the same. Massage strength should be changed from light to heavy gradually with a moderate rate. Besides, the vertical tension of the surgical incision should not be increased.

Part 3	Kegel motion	Specific methods were the same as those for the control group, and the exercise was performed 5 times.

Part 4	Cross-leg anus lifting motion	Patients were asked to remain decubitus or in the standing position and keep thighs crossed. Besides, perinaeum needed to be clamped by hips and thighs, and the muscles around anus needed to be tightened and lifted upward slowly and gradually. The above actions should be kept for 5 seconds, and then patients were allowed to relax for 10 seconds. The group of exercise was performed 5 times.

Part 5	Bridging anus lifting motion	Patients were asked to lie on their backs in bed with their knees bent and the soles of their feet pushing the bed. With heads, elbows, and feet as the supporting points, hips were lifted by pelvic floor muscles, and hip muscles, and perineal muscles were contracted. Patients needed to try their best to keep the above actions for 5 seconds, and then they were allowed to lower their hips and relax for 5 seconds. The group of exercises was performed 5 times.

Part 6	Leg motion	Tsusanli was pressed and kneaded for 1 minute with the thumbs.
		When the acupuncture points become swollen and get a fever, the degree of pressure should remain the same. After that, two legs were lifted in turns. Besides, the thighs were kept at a 90° angle to the bodies. With a good physical condition, two legs could be gradually lifted, which should be repeated 5 times.

**Table 2:** MRI examination scanning parameters.

Sequence	Position	Time of repetition (TR)	Time of echo (TE)	Slice thickness/slice spacing	Matrix	Fat suppression
T2WI	Sagittal position	4400	80	4/0.9	330^*∗*^330	Yes
T2WI	Axial position	4900	85	4/0.9	330^*∗*^330	Yes
T2WI	Axial position	4900	80	4/0.9	330^*∗*^330	No
T1WI	Axial position	673	23	4/0.9	330^*∗*^330	Yes
T2WI	Coronal position	4100	95	4/0.9	330^*∗*^330	No

**Table 3:** General data on patients in two groups.

Items	Experimental group (*n* = 44)	Control group (*n* = 44)	Statistical values	*P*
Age (years old)	53.1 ± 10.5	55.8 ± 11.6	0.612	0.731
Gender (case)	—	—	0.044	0.939
Male	23 (52%)	18 (41%)	—	—
Female	21 (48%)	26 (59%)	—	—
Tumor level (case)	—	—	2.886	0.544
High differentiation	15 (34%)	10 (23%)	—	—
Moderate differentiation	20 (45%)	26 (59%)	—	—
Low differentiation	9 (20%)	8 (18%)	—	—
Anal edge tumor height	8.2 ± 2.6	7.3 ± 3.1	−1.127	0.485

## Data Availability

The data used to support the findings of this study are available from the corresponding author upon request.
